The article "Evaluation of Antiarthritic and Antinociceptive Effects of Cedrol in a Rat Model of Arthritis" was published in 2022. Journal: Oxid Med Cell Longev.

# Evaluation of Antiarthritic and Antinociceptive Effects of Cedrol in a Rat Model of Arthritis

**DOI:** 10.1155/2022/4943965

**Published:** 2022-04-25

**Authors:** Fatemeh Forouzanfar, Ali Mohammad Pourbagher-Shahri, Hamed Ghazavi

**Affiliations:** ^1^Neuroscience Research Center, Mashhad University of Medical Sciences, Mashhad, Iran; ^2^Department of Neuroscience, Faculty of Medicine, Mashhad University of Medical Sciences, Mashhad, Iran; ^3^Medical Toxicology Research Center, Faculty of Medicine, Mashhad University of Medical Sciences, Mashhad, Iran

## Abstract

Pharmacological studies revealed that cedrol, a natural sesquiterpene, has antioxidant, anti-inflammatory, and analgesic properties. This study is aimed at evaluating the potential antiarthritic activity of cedrol in a rat experimental model of arthritis induced by using complete Freund's adjuvant (CFA). Arthritis was induced in Wistar rats by CFA (0.1 ml) injection. Cedrol (10 and 20 mg/kg) and indomethacin (5 mg/kg) were orally administered from day one and continued for 21 days. The antiarthritic activity was assessed through mechanical allodynia and thermal hyperalgesia responses, paw edema assessment, and arthritis scores. Serum TNF-*α* and IL-1*β* levels were measured for the evaluation of inflammation. Furthermore, serum oxidative stress markers, including malondialdehyde (MDA) and thiol levels, as well as superoxide dismutase (SOD) and glutathione peroxidase (GPx) activities, were also assessed. Oral administration of cedrol and indomethacin significantly decreased paw edema and arthritis score. Besides, cedrol and indomethacin significantly decreased pain responses. In the serum of the CFA group, TNF-*α*, IL-1*β*, and MDA were higher, while thiol and SOD and GPx were lower than the control group. Treatment by cedrol and indomethacin corrected the biochemical parameters in the serum. In this study, cedrol offers potential antiarthritic properties through its anti-inflammatory and antioxidant effects.

## 1. Introduction

Rheumatoid arthritis (RA) is a chronic systemic inflammatory disease described by multijoint inflammation, pain, and destruction of cartilage and bone [1, 2]. The disease may progress to a severe disability with negative consequences on the quality of life and increased mortality rate [3]. Autoimmunity and chronic inflammation are activated by an imbalance between pro- and anti-inflammatory cytokines, resulting in joint damage in RA [4]. Although nonsteroidal anti-inflammatory drugs effectively reduce symptoms, they do not prevent the disease from progressing and do not protect the tissue or joint against erosion. Also, they have severe side effects or cardiovascular complications; growing interest in herbal remedies in RA patients indicates the need to find new agents from herbal medicines [5]. Indeed, safe and effective agents for the treatment of RA are urgently required. Natural plant compounds are suggested to prevent or treat RA [6]. Terpenes, also known as terpenoids, are the largest and most diverse group of natural products. They are classified according to the number of isoprene units to mono, di, tri, tetra, and sesquiterpenes [7]. Sesquiterpenes (C15) are composed of 3 units of isoprenoid, which are secondary metabolites produced mostly in plants [8]. Recent studies showed that sesquiterpenes have various therapeutic effects, such as being effective in pain management [9], protection against stroke [10], and RA [11]. Cedrol, a natural sesquiterpene, is known to carry many pharmacological effects, including antioxidant [12], anti-inflammatory [13], antibacterial [14], analgesic [12], sedative [15], hair growth inducer [16], platelet-activating factor (PAF) antagonist [17], and antitumor effects [18]. The present investigation is aimed at evaluating the potential antiarthritic effect of cedrol on complete Freund's adjuvant- (CFA-) induced experimental arthritis in rats.

## 2. Chemicals

Ketamine and xylazine were bought from Alfasan Pharmaceutical Co. (Woerden, Netherlands). Pyrogallol, 2-thiobarbituric acid (TBA), CFA, dimethyl sulfoxide (DMSO), potassium chloride, hydrochloric acid (HCl), trichloroacetic acid (TCA), cedrol, and ethylenediaminetetraacetic acid (EDTA) were purchased from Sigma-Aldrich (Sigma-Aldrich, St. Louis, MO).

## 3. Animals

Adult male rats weighing between 180 and 220 g were provided by the animal facility of the medical school, Mashhad University of Medical Sciences (MUMS), Mashhad, Iran. Animals were kept at 22-25°C with food and water ad libitum with a natural dark and light (12: 12 h) cycle. All experiments were conducted according to the care and use of Laboratory Animals and Animal Ethics Guidelines of MUMS.

## 4. Induction of Arthritis and Treatment Protocol

Arthritis was induced on day 0 by a 0.1 ml subcutaneous injection of CFA into the right hind footpad of the rat. Rats were randomly divided into five experimental groups.

- *Group I*. For the control group, rats were administered with 0.1 ml normal saline instead of CFA in the right hind paw
- *Group II*. For the CFA group, rats were administered with 0.1 ml CFA
- *Group III*. For the positive control group, rats were administered with indomethacin (5 mg/kg, p.o.) daily for 21 days after the CFA injection
- *Group IV*. For the drug-treated group, rats were administered with cedrol (10 mg/kg, p.o.) daily for 21 days after the CFA injection
- *Group V*. For the drug-treated group, rats were administered with cedrol (20 mg/kg, p.o.) daily for 21 days after the CFA injection

### 4.1. Drug Administration

All drugs/vehicles were precisely administered by oral gavage. Cedrol dissolved in saline containing 1% DMSO. All measurements were performed blinded, and the investigator did not know what treatment each rat received.

Nociceptive behavioral examines, paw volume evaluation, and arthritis score were examined on days 0, 7, 14, and 21. The hind footpad's paw thickness (right) was measured in each rat using a caliper.

### 4.2. Arthritis Score

The severity of arthritis was assessed as follows [1]: 0 = no change, 1 = mild erythema or swelling of the digits, 2 = moderate swelling and erythema, 3 = severe swelling and erythema involving the ankle, and 4 = ankylosis and inability to bend the ankle.

### 4.3. Thermal Hyperalgesia

The hot plate was used to assess thermal hyperalgesia. In this test, rats were individually placed on a hot plate maintained at 55°C. The latency to the first sign of paw licking or jump response to avoid the heat nociception was taken as an index of the pain threshold; the cut-off time was set at 10 s to prevent any injury to the tissues of the paws [1].

### 4.4. Mechanical Allodynia

Animals were placed on an elevated box (30 × 30 × 30 cm) with a metal wire floor, and an ascending series of von Frey filaments (Bioseb) were applied in ascending style to the plantar surface. The cut-off threshold was set at 60 g to prevent tissue damage. Each filament was tested five times. A positive response is if the animal responded to at least three withdrawals out of five consecutive trials. That gram force was considered as the paw withdrawal threshold [19].

### 4.5. Biochemical Assays

The serum interleukin 1 *β* (IL-1*β*) and tumor necrosis factor *α* (TNF-*α*) levels were detected using a commercial ELISA kit (Karmania Pars Gene Company, Kerman, Iran). The levels of malondialdehyde (MDA), as the final product of the lipid peroxidation process, superoxide dismutase (SOD) activity, and thiol concentration in serum, were assessed based on the methods reported by previous publication [20]. Glutathione peroxidase (GPX) activity was detected using a commercial ELISA GPX assay kit (ZellBio, German).

### 4.6. Statistical Analysis

GraphPad Prism (version 6.0) was used for analyzing the data. All data were shown as mean ± SEM. Behavioral parameters were measured by two-way analysis of variance (ANOVA) followed by Bonferroni's test. Biochemical parameters were measured by one-way ANOVA followed by Tukey's test. *p* values lower than 0.05 were statistically significant.

## 5. Results

### 5.1. Effect of Cedrol on the Arthritis Score in CFA-Induced Arthritic Rats

As shown in Figure 1, the arthritis score in all groups on day 0 was 0. The arthritis score in the cedrol (10 mg/kg) group was lower than that detected in the CFA group on day 21 (*p* < 0.05). The arthritis score in the cedrol (20 mg/kg) group was lower than that detected in the CFA group on days 7, 14, and 21 (*p* < 0.05, *p* < 0.001, and *p* < 0.001, respectively). A significant decrease in arthritic index was recorded in the indomethacin group compared to the CFA group on days 7, 14, and 21 (*p* < 0.05, *p* < 0.01, and *p* < 0.001, respectively).

### 5.2. Effect of Cedrol on Paw Volume in CFA-Induced Arthritic Rats

As shown in Figure 2, there was no significant difference in paw volume between groups on day 0. The paw volume in the CFA group significantly increased on days 7, 14, and 21 compared to the control group (*p* < 0.001). The paw volume in the indomethacin (5 mg/kg) group was lower than that detected in the CFA group on day 7 (*p* < 0.01). The paw volume in the cedrol (20 mg/kg) group and indomethacin (5 mg/kg) group was lower than that detected in the CFA group on day 14 (*p* < 0.05 and *p* < 0.01, respectively). Over time, the paw volume decreased further in the treatment groups; the paw volume in the cedrol (20 mg/kg) and indomethacin (5 mg/kg) group was lower than that detected in the CFA group on day 21 (*p* < 0.01).

### 5.3. Effect of Cedrol on Thermal Hyperalgesia in CFA-Induced Arthritic Rats

The CFA-injected rats showed a significant decrease in thermal hyperalgesia threshold on day 7, continuing until day 21 compared to the control group (*p* < 0.001). However, highest dose of cedrol (20 mg/kg) attenuated CFA-induced thermal hyperalgesia on days 7, 14, and 21 compared to the CFA-control group (*p* < 0.05, *p* < 0.01, and *p* < 0.01, respectively). Indomethacin (5 mg/kg) attenuated CFA-induced thermal hyperalgesia on days 14 and 21 compared to the CFA-control group (*p* < 0.05). 10 mg/kg cedrol treatment also led to a significant improvement on day 21 (increased paw withdrawal latency) compared to the CFA-control group (*p* < 0.05) (Figure 3).

### 5.4. Effect of Cedrol on Mechanical Allodynia in CFA-Induced Arthritic Rats

CFA-injected rats showed a significant reduction in paw withdrawal mechanical threshold (mechanical allodynia) on days 7, 14, and 21 as compared with the nonarthritic control group, which continued to worsen till the end of the experiment (*p* < 0.001). However, treatment with cedrol (10 mg/kg) did not significantly differ from CFA-treated rats. Cedrol (20 mg/kg) showed a statistically significant enhancement in paw withdrawal threshold in CFA-induced arthritic rats on days 7, 14, and 21 compared to the CFA-control group (*p* < 0.05, *p* < 0.01, and *p* < 0.01, respectively). Similarly, indomethacin (5 mg/kg) also significantly augmented the paw withdrawal threshold in the CFA group on days 7, 14, and 21 compared to the CFA-control group (*p* < 0.05, *p* < 0.05, and *p* < 0.01, respectively) (Figure 4).

### 5.5. Effect of Cedrol on the Serum Levels of IL-1*β* and TNF-*α* in CFA-Induced Arthritic Rats

The IL-1*β* level was significantly higher (*p* < 0.001) in the CFA group compared to the control group. The treatment with indomethacin was effective in decreasing IL-1*β* level in serum of CFA-induced rats compared to the CFA-control group (*p* < 0.01), besides the treatment with cedrol (20 mg/kg) reduced IL-1*β* level in serum of CFA-induced rats compared to the CFA-control group (*p* < 0.01) (Figure 5(a)).

As displayed in Figure 5(b), administration of CFA significantly increased the serum TNF-*α* level (*p* < 0.001) in the arthritic (CFA group) compared to the control group. The treatment with indomethacin was effective to decrease TNF-*α* level in serum of CFA-induced rats (*p* < 0.01 versus CFA group), besides the treatment with cedrol (10 and 20 mg/kg) reduced TNF-*α* level in serum of CFA-induced rats compared to the CFA group (*p* < 0.05 and *p* < 0.01, respectively).

### 5.6. Effect of Cedrol on the Oxidative Stress in CFA-Induced Arthritic Rats

MDA level was significantly higher (*p* < 0.001) in the arthritic (CFA group) compared to the control group. The treatment with indomethacin was effective in decreasing MDA level in serum of CFA-induced rats compared to the CFA group (*p* < 0.05), besides the treatment with cedrol (20 mg/kg) reduced MDA level in serum of CFA-induced rats compared to the CFA-control group (*p* < 0.05) (Figure 6(a)).

As shown in Figure 6(b), administration of CFA markedly decreased serum levels of thiol as compared to the control group (*p* < 0.01). The treatment with cedrol (20 mg/kg) and indomethacin significantly increased thiol level in serum of CFA-induced rats compared to the CFA-control group (*p* < 0.01).

SOD activity was significantly lower (*p* < 0.001) in the arthritic (CFA group) compared to the control group. In the treatment groups (cedrol (20 mg/kg) and indomethacin), SOD activity elevated significantly compared to the CFA group (*p* < 0.01) (Figure 6(c)).

Gpx activity was significantly lower (*p* < 0.01) in the arthritic (CFA group) compared to the control group. The treatment with indomethacin was effective to increase Gpx activity in serum of CFA-induced rats compared to the CFA-control group (*p* < 0.05), besides the treatment with cedrol (20 mg/kg) increased Gpx activity in serum of CFA-induced rats compared to the CFA group (*p* < 0.05) (Figure 6(d)).

## 6. Discussion

The CFA-induced experimental model of arthritis is known to have numerous human RA features, such as robust hypersensitivity to mechanical and heat stimuli, polyarticular inflammation, and deterioration of the joint structures. This model is widely used to study RA's pathogenesis and assess potential therapeutic targets useful for the treatment of RA [1, 21, 22]. Following intraplantar injection of CFA, the mycobacterial constituents in the CFA cause T-lymphocytes to provoke a robust immune response in the rat paws. The T-lymphocytes interact with dendritic cells, monocytes, and macrophages to produce the major proinflammatory cytokine participating in the pathogenesis of RA, including TNF-*α*, IL-1*β*, and IL-6 in the synovial membrane [23–26]. The interaction between these proinflammatory mediators causes synovial inflammation and cartilage/bone destruction [27]. It has been revealed that TNF-*α* blockade reduces the symptoms of RA [28]. The inflammatory cytokines IL-1*β* and TNF-*α* are the therapeutic targets in RA treatment strategies [29, 30].

On the other hand, arthritis can cause chronic inflammatory pain. Moreover, chronic inflammatory pain is modeled via CFA attributed to provoke inflammatory cytokines, which sensitizes nociceptive neurons and reduces the pain threshold [31]. Previous studies have highlighted that sesquiterpenes show anti-inflammatory, antioxidant [32], and analgesic properties [33]. Consequently, in the present study, the potential protective properties of cedrol were examined against CFA-induced arthritis in rats. According to the present study, cedrol improved the nociception behaviors of the rats exposed to CFA. Anti-inflammatory and antioxidant effects also accompanied it. Cedrol reduced the paw's thickness by inhibiting the release of inflammatory mediators (IL-1B and TNF-*α*), indicating its anti-inflammatory potential in CFA-induced arthritis. As a nonsteroidal anti-inflammatory drug, indomethacin inhibits the production of prostaglandins by inhibiting the activity of cyclooxygenase [34]. In this study, indomethacin reduced the thickness of the paw and exerted antinociceptive behaviors. Besides, indomethacin reduced serum levels of TNF-*α* and IL-1*β* as well. Antioxidant therapy has thus represented an effective treatment for oxidative stress/inflammation-related diseases. Oxidative stress occurs due to an imbalance between prooxidants and antioxidants and consequent excessive production of reactive oxygen species (ROS) [35]. Several defense systems, including enzymatic (SOD and GPx) and nonenzymatic antioxidants (GSH), have been involved in the cells preventing uncontrolled ROS. Indeed, these antioxidants' impairments have been reported in active RA patients [36]. ROS production inside the joints has an essential role in arthritis pathogenesis since oxidants by direct action or indirect activation of latent collagenases degrade matrix ingredients [37]. Besides, ROS are positively linked with the severity of RA [38]. ROS participate in the signaling of inflammation. Mitochondrial ROS stimulate proinflammatory cytokine production, IL-1B, IL-6, and TNF-*α*.

On the other hand, the inflammation process also causes oxidative stress as host immune cells, like neutrophils, also known as polymorphonuclear neutrophils, release large amounts of ROS via the NADPH oxidase enzyme pathway [38]. In the current study, cedrol or indomethacin showed antioxidant properties, as it decreased the MDA levels while antioxidant molecules (thiol, SOD, and GPx) increased. These results are in accordance with the previous study reported that administration of cedrol (20 and 40 mg/kg, i.p.) once a day for 14 days postchronic constriction injury model of neuropathic pain attenuated nociception pain behaviors in rats by inhibition of inflammatory response and reduction of oxidative stress markers [12]. Another study showed cedrol reduced collagen-induced arthritis in mice and modulates the inflammatory response in lipopolysaccharide-mediated fibroblast-like synoviocytes [39]. Treatment with Budlein A, a sesquiterpene lactone from *Viguiera robusta*, showed anti-inflammatory and analgesic effects in antigen-induced arthritis in mice [40]. Arthritis score and swelling of the paw are indexes to access the antiarthritic action of numerous medicines [5], and these indexes were used to evaluate the effect of cedrol in this study. The cedrol groups noteworthy attenuated paw thickness and arthritis scores. In the current investigation, cedrol modified different parameters of arthritis in rats, including arthritic score, paw volume, nociception behaviors, oxidative stress markers, and inflammation. Thus, cedrol may be effective as a long-term antiarthritis agent to overcome the distressing manifestation of RA.

In conclusion, we conclude that cedrol exhibits antiarthritic properties presumably through inhibition of oxidative stress and inflammation. Overall, these results provided supportive evidence for the therapeutic potential of cedrol in RA treatment.

## Figures and Tables

**Figure 1:** Effects of cedrol on arthritis score. Values are mean ± SEM, *n* = 8 in each group. ^∗^*p* < 0.05, ^∗∗^*p* < 0.01, and ^∗∗∗^*p* < 0.001 vs. CFA group.

**Figure 2:** Effects of cedrol on paw volume. Values are mean ± SEM, *n* = 8 in each group. ^∗^*p* < 0.05 and ^∗∗^*p* < 0.01 vs. CFA group. ###*p* < 0.001 vs. control group.

**Figure 3:** Effect of cedrol on paw withdrawal latency (s). Values are mean ± SEM. *n* = 8 in each group. ^∗^*p* < 0.05 and ^∗∗^*p* < 0.01 vs. CFA group. ###*p* < 0.001 vs. control group.

**Figure 4:** Effect of cedrol on paw withdrawal threshold (g). Values are mean ± SEM. *n* = 8 in each group. ^∗^*p* < 0.05 and ^∗∗^*p* < 0.01 vs. CFA group. ###*p* < 0.001 vs. control group.

**Figure 5:** Effect of cedrol on (a) IL-1*β* and (b) TNF-*α* concentration. Values are mean ± SEM. *n* = 6 in each group. ^∗^*p* < 0.05 and ^∗∗^*p* < 0.01 vs. CFA group. ###*p* < 0.001 vs. control group.

**Figure 6:** Effect of cedrol on (a) MDA concentration, (b) thiol concentration, (c) SOD activity, and (d) Gpx activity. Values are mean ± SEM. *n* = 6 in each group. ^∗^*p* < 0.05 and ^∗∗^*p* < 0.01 vs. CFA group. ##*p* < 0.001 and ###*p* < 0.001 vs. control group.

## Data Availability

The dataset that supports the results and findings of this research is available from the corresponding author upon request.

## References

[1] Kumar A., Dhaliwal N., Dhaliwal J., Dharavath R. N., Chopra K. (2020). Astaxanthin attenuates oxidative stress and inflammatory responses in complete Freund-adjuvant-induced arthritis in rats. *Pharmacological Reports*.

[2] Nasuti C., Fedeli D., Bordoni L. (2019). Anti-inflammatory, anti-arthritic and anti-nociceptive activities of Nigella sativa oil in a rat model of arthritis. *Antioxidants*.

[3] Mahdi H. J., Khan N. A. K., Asmawi M. Z. B., Mahmud R., Vikneswaran A., Murugaiyah L. (2018). *In vivo* anti-arthritic and anti-nociceptive effects of ethanol extract of *Moringa oleifera* leaves on complete Freund's adjuvant (CFA)-induced arthritis in rats. *Integrative medicine research*.

[4] McInnes I. B., Schett G. (2007). Cytokines in the pathogenesis of rheumatoid arthritis. *Nature Reviews Immunology*.

[5] Tong Z., Cheng L., Song J. (2018). Therapeutic effects of Caesalpinia minax Hance on complete Freund’s adjuvant (CFA)-induced arthritis and the anti-inflammatory activity of cassane diterpenes as main active components. *Journal of Ethnopharmacology*.

[6] Lindler B. N., Long K. E., Taylor N. A., Lei W. (2020). Use of herbal medications for treatment of osteoarthritis and rheumatoid arthritis. *Medicine*.

[7] Cox-Georgian D., Ramadoss N., Dona C., Basu C. (2019). *Therapeutic and Medicinal Uses of Terpenes*.

[8] Bártíková H., Hanusova V., Skalova L., Ambroz M., Bousova I. (2014). Antioxidant, pro-oxidant and other biological activities of sesquiterpenes. *Current topics in medicinal chemistry*.

[9] Aguilar-Ávila D. S., Flores-Soto M. E., Tapia-Vázquez C., Pastor-Zarandona O. A., López-Roa R. I., Viveros-Paredes J. M. (2019). *β*-Caryophyllene, a natural sesquiterpene, attenuates neuropathic pain and depressive-like behavior in experimental diabetic mice. *Journal of medicinal food*.

[10] Yousefi-Manesh H., Dehpour A. R., Shirooie S. (2021). Isofuranodiene, a natural sesquiterpene isolated from wild celery (*Smyrnium olusatrum* L.), protects rats against acute ischemic stroke. *Pharmaceuticals*.

[11] Gao S., Wang Q., Tian X.-H. (2017). Total sesquiterpene lactones prepared from *Inula helenium* L. has potentials in prevention and therapy of rheumatoid arthritis. *Journal of Ethnopharmacology*.

[12] Sakhaee M. H., Sayyadi S. A. H., Sakhaee N. (2020). Cedrol protects against chronic constriction injury-induced neuropathic pain through inhibiting oxidative stress and inflammation. *Metabolic Brain Disease*.

[13] Jantan I., Rafi I., Jalil J. (2005). Platelet-activating factor (PAF) receptor-binding antagonist activity of Malaysian medicinal plants. *Phytomedicine*.

[14] Oh I., Yang W.-Y., Park J. (2011). In vitro Na+/K+-ATPase inhibitory activity and antimicrobial activity of sesquiterpenes isolated from Thujopsis dolabrata. *Archives of pharmacal research*.

[15] Kagawa D., Jokura H., Ochiai R., Tokimitsu I., Tsubone H. (2003). The sedative effects and mechanism of action of cedrol inhalation with behavioral pharmacological evaluation. *Planta Medica*.

[16] Zhang Y., Han L., Chen S.-S., Guan J., Qu F.-Z., Zhao Y.-Q. (2016). Hair growth promoting activity of cedrol isolated from the leaves of Platycladus orientalis. *Biomedicine & Pharmacotherapy*.

[17] Yang H. O., Suh D.-Y., Han B. H. (1995). Isolation and characterization of platelet-activating factor receptor binding antagonists from Biota orientalis. *Planta Medica*.

[18] Loizzo M., Tundis R., Menichini F., Saab A., Statti G., Menichini F. (2008). Antiproliferative effects of essential oils and their major constituents in human renal adenocarcinoma and amelanotic melanoma cells. *Cell Proliferation*.

[19] Forouzanfar F., Hosseinzadeh H., Khorrami M. B., Asgharzade S., Rakhshandeh H. (2019). Attenuating effect of Portulaca oleracea extract on chronic constriction injury induced neuropathic pain in rats: an evidence of anti-oxidative and anti-inflammatory effects. *CNS & Neurological Disorders-Drug Targets (Formerly Current Drug Targets-CNS & Neurological Disorders)*.

[20] Khorrami M. B., Sadeghnia H. R., Pasdar A. (2019). Antioxidant and toxicity studies of biosynthesized cerium oxide nanoparticles in rats. *International Journal of Nanomedicine*.

[21] Bendele A. (2001). Animal models of rheumatoid arthritis. *Journal of Musculoskeletal & Neuronal Interactions*.

[22] Lal R., Dhaliwal J., Dhaliwal N., Dharavath R. N., Chopra K. (2021). Activation of the Nrf2/HO-1 signaling pathway by dimethyl fumarate ameliorates complete Freund’s adjuvant-induced arthritis in rats. *European Journal of Pharmacology*.

[23] Voon F.-L., Sulaiman M. R., Akhtar M. N. (2017). Cardamonin (2′, 4′-dihydroxy-6′-methoxychalcone) isolated from *Boesenbergia rotunda* (L.) Mansf. inhibits CFA-induced rheumatoid arthritis in rats. *European journal of pharmacology*.

[24] Tran C. N., Lundy S. K., Fox D. A. (2005). Synovial biology and T cells in rheumatoid arthritis. *Pathophysiology*.

[25] Magyari L., Varszegi D., Kovesdi E. (2014). Interleukins and interleukin receptors in rheumatoid arthritis: research, diagnostics and clinical implications. *World Journal of Orthopedics*.

[26] Qin F., Zhang H., Liu A. (2019). Analgesic effect of *Zanthoxylum nitidum* extract in inflammatory pain models through targeting of ERK and NF-*κ*B signaling. *Frontiers in pharmacology*.

[27] He P., Hu Y., Huang C. (2020). N-Butanol extract of *Gastrodia elata* suppresses inflammatory responses in lipopolysaccharide-stimulated macrophages and complete Freund’s adjuvant-(CFA-) induced arthritis rats via inhibition of MAPK signaling pathway. *Evidence-Based Complementary and Alternative Medicine*.

[28] Mewar D., Wilson A. G. (2011). Treatment of rheumatoid arthritis with tumour necrosis factor inhibitors. *British journal of pharmacology*.

[29] Zhuang Y., Lyn S., Lv Y. (2013). Pharmacokinetics and safety of golimumab in healthy Chinese subjects following a single subcutaneous administration in a randomized phase I trial. *Clinical drug investigation*.

[30] Nikfar S., Saiyarsarai P., Tigabu B. M., Abdollahi M. (2018). Efficacy and safety of interleukin-1 antagonists in rheumatoid arthritis: a systematic review and meta-analysis. *Rheumatology international*.

[31] Liu T., Su B. (2021). *Styphnolobium japonicum* (L.) Schott flower extract alleviates oxidative stress and inflammatory factors in the adjuvant-induced arthritis rat model. *Research*.

[32] Dahham S. S., Tabana Y. M., Iqbal M. A. (2015). The anticancer, antioxidant and antimicrobial properties of the sesquiterpene *β*-caryophyllene from the essential oil of Aquilaria crassna. *Molecules*.

[33] Chavan M. J., Wakte P. S., Shinde D. B. (2012). Analgesic and anti-inflammatory activities of the sesquiterpene fraction from *Annona reticulata* L. bark. *Natural product research*.

[34] Nalamachu S., Wortmann R. (2014). Role of indomethacin in acute pain and inflammation management: a review of the literature. *Postgraduate Medicine*.

[35] Mititelu R. R., Pădureanu R., Băcănoiu M. (2020). Inflammatory and oxidative stress markers—mirror tools in rheumatoid arthritis. *Biomedicine*.

[36] Quiñonez-Flores C. M., González-Chávez S. A., Del Rio N. D., Pacheco-Tena C. (2016). Oxidative stress relevance in the pathogenesis of the rheumatoid arthritis: a systematic review. *BioMed research international*.

[37] Vasanthi P., Nalini G., Rajasekhar G. (2009). Status of oxidative stress in rheumatoid arthritis. *International journal of rheumatic diseases*.

[38] García-Sánchez A., Miranda-Díaz A. G., Cardona-Muñoz E. G. (2020). The role of oxidative stress in physiopathology and pharmacological treatment with pro- and antioxidant properties in chronic diseases. *Oxidative Medicine and Cellular Longevity*.

[39] Chen X., Shen J., Zhao J.-m. (2020). Cedrol attenuates collagen-induced arthritis in mice and modulates the inflammatory response in LPS-mediated fibroblast-like synoviocytes. *Food & Function*.

[40] Zarpelon A. C., Fattori V., Souto F. O. (2017). The sesquiterpene lactone, budlein A, inhibits antigen-induced arthritis in mice: role of NF-*κ*B and cytokines. *Inflammation*.

